# Diagnosing Cancer Using IOT and Machine Learning Methods

**DOI:** 10.1155/2022/9896490

**Published:** 2022-05-28

**Authors:** Mohammed Maray, Mohammed Alghamdi, Malik Bader Alazzam

**Affiliations:** ^1^College of Computer Science, King Khalid University, Abha 62529, Saudi Arabia; ^2^Jeddah University, Jeddah, Saudi Arabia; ^3^Information Technology College, Ajloun National University, Jordan

## Abstract

Breast cancer affects one in every eight women and is the most common cancer. *Aim*. To diagnose breast cancer, a potentially fatal condition, using microarray technology, large datasets can now be used. *Methods*. This study used machine learning algorithms and IOT to classify microarray data. They were created from two sets of data: one with 1919 protein types and one with 24481 protein types for 97 people, 46 of whom had a recurring disease and 51 of whom did not. The apps were written in Python. Each classification algorithm was applied to the data separately, without any feature elimination or size reduction. Second, two alternative feature reduction approaches were compared to the first case. In this case, machine learning techniques like Adaboost and Gradient Boosting Machine are used. *Results*. Before applying any feature reduction techniques, the logistic regression method produced the best results (90.23%), while the Random Forest method produced good results (67.22%). In the first data, SVM had the highest accuracy rate of 99.23% in both approaches, while in the second data, SVM had the highest rate of 87.87% in RLR and 88.82% in LTE. Deep learning was also done with MLP. The relationship between depth and classification accuracy was studied using it at various depths. After a while, the accuracy rate declined as the number of layers increased. The maximum accuracy rate in the first data was 97.69%, while it was 68.72% in the second. As a result, adding layers to deep learning does not improve classification accuracy.

## 1. Introduction

Cancer is a disease that consists of the uncontrolled proliferation of cells in various organs and ranks second among the causes of death in Arabic countries [1]. Breast cancer is the most common type of cancer among women and causes the most deaths. Breast cancer is the first among the cancer types seen in women, and there is a risk of developing this cancer in one out of every eight women in a lifetime. Diagnosis at an early stage increases the chances of successful treatment and survival of the patient. Microarray technology offers a tremendous opportunity to detect the relationship between diseases and genes. Having too many features here makes it difficult to analyze this data. Not all of these features are related to the disease in question, and the elimination of these irrelevant features makes it difficult to find genes associated with the disease. At this point, feature reduction methods come into play. Elimination of the most unrelated genes generally increases the classification accuracy. The main application areas of machine learning are artificial intelligence and data mining. Data mining is selecting useful data from a database for use in learning. For example, a doctor uses necessary information from the patient's previous medical files to prescribe to a patient, or selecting transactions from past transactions will provide evidence in understanding credit card fraud [2, 3]. On the other hand, artificial intelligence needs model creation by machine learning such as robotics, image processing, computer vision, and recognition of objects in images. Machine learning relies on building a general model from real-life data [4]. With this model, it is aimed to know how to behave when faced with new data. For example, a chess player gains experience and takes steps based on these experiences. The machine also makes a decision based on its experience. Classification is the process of grouping datasets by looking at certain properties. Using this data, the goal is to find features that relate them to each other. We divide these data into two groups: training and test data. Training data are images, attributes, and databases used to create a learning model. Test data are data applied to test the model. With technological advances, collecting data has become easier. These data are frequently used in medicine and other fields. Many studies analyze large amounts of data to help experts diagnose the disease causes. The data from these microarrays are analyzed to extract useful information or create a model from which we can structure and thus benefit from the information they contain. Many previous articles and theses use them to classify or predict. A model is created that can predict for two-class supervised learning. Many studies that we will discuss in the literature review section use classical machine learning methods. Supervised and unsupervised machine learning has recently been applied to gene expression data. These methods use class labels to identify data classes. It is also used to classify cancer patients. This is vital for patients [3, 5]. This study divided data into the study and test groups. It is divided into two groups, one sick and one healthy, with 68 people in each. The 5-fold crossover method was used to test SVM, K-FCV, and Random Forest algorithms, with SVM providing the best results. So, SVM classified 98% of the study data and 100% of the test data correctly. Again, our dataset has been used before [6, 7]. Abhineet Gupta et al. selected the best 130, 99, and 102 features. Naive Bayes achieved 89 percent with ReliefF feature selection and 84 percent with SVM-SME feature elimination. The k-S test outperformed the Wilcoxon and *T*-Test methods (Su et al.) [5]. Then, we compared the k-S test to other CFS feature selection methods. Except for ReliefF and mRMR, all CFS and k-S Test selection methods are compared. All were compared using SVM. The rates are 80.5, 87.4, 82.4, 59.4, and 788. The C4.5 decision tree method outperformed Naive Bayes (95.79%) by 97.9%. Endo et al. This study estimated 37,256 patients' 5-year survival rates. The Logistic Regression algorithm got the best result with 85.8% [8, 9]. However, leaving too few features appears to increase variance. The min-max model selection criterion was applied. Algorithms like SVM and Weighted Voting were used to compare LOO and error rate. This method had the least error in all datasets. It had three times less error in the other. All LOO and min-max comparisons with varying numbers of data had less error.

## 2. Materials and Methods

### 2.1. Materials

The data studied in this work are the numerical NumPy library of the Python language, which is used to process multidimensional data such as matrix arrays and enables us to apply mathematical operations to these data. Pandas library that allows us to structure data, Scikit-learn library which contains machine learning classification, regression, and clustering algorithms, and Keras library which provides deep learning application were used. The first amount of the data used was the data from the study [2, 10], which included 1927 features from 133 individuals, 11 of whom were healthy and 122 of whom were patients. The other set from the study (Yersal and Barutca) [11], 46 of whom had a breast cancer recurrence, contains 24481 features belonging to 97 individuals, 51 of which are not. These data are in a matrix with 133 rows and 1919 columns. Our other data consist of 97 rows and 24481 columns. In our first data, coding was made as patients and nonpatients. These data are divided into two groups for training and testing. The machine is trained with the training group, and the classification performance is tested with the test group.

### 2.2. Methodology-Machine Learning Methods

#### 2.2.1. Logistic Regression Algorithm

The basis of logistic regression, a classification algorithm, is based on the “sigmoid function.” The reason for using the sigmoid function in this algorithm is to obtain a value between 0 and 1 as an output value. Logistic regression is formed by adding the sigmoid function to the linear function (*x*)=*w*^*T*^*x*+*b*. If we say *z*=*f*(*x*), from equation (1), (*z*) equals a value between 0 and 1, regardless of the real number of variable *z*.

(1) $$\begin{array}{c} \sigma \left(z\right)=\frac{1}{1}+e^{-z}. \end{array}$$

#### 2.2.2. *K*-Nearest Neighborhood Algorithm (kNN)

It is one of the simplest algorithms. The working principle is as follows: a sample is in the class of its *k*-nearest neighbors. It is in the class of its nearest neighbor if *k* is 1. The Euclidean distance is commonly used to calculate proximity. The *k* number is crucial in this technique since it decides the class in which our sample will be included. Also, if the categorization is equal, it is impossible to tell which class *k* will be included. The finest results usually come from 1.3 or 5. The algorithm divides the data into training and test. A sample dataset is classified by calculating its distance from each training data set in the feature space. It verifies which classes the nearest neighbors belong to, up to *k*. Sample data are included in the majority class. The *k* value and the distance calculation method affect the performance of this algorithm.

#### 2.2.3. Decision Trees

Decision trees are utilized in numerous fields, including character recognition and medicine. It works by reducing a complex operation to a series of simple decisions. This simplifies the problem's interpretation. A model consisting of one or more trees is constructed using tagged input data. This model then guesses the class of unknown data. Attributes are values in data. Any type of value can be used here. The decision tree starts at the root node. This node has no entry. Test nodes are intermediates. The leaves are the decision nodes. An intermediate node in a decision tree divides the sample space (dataset) into two or more subspaces. After all operations, the leaves, or last nodes, are assigned the best values. The outputs of these procedures are used to classify data from root to leaf. It is a simple approach to comprehend.

#### 2.2.4. Random Forest

This method employs many trees instead of a decision tree. A random vector determines the value of each tree in the forest [12, 13]. The number of trees can be planned. Each decision tree's training data are unique. The optimum feature selection in each tree is made by comparing randomly generated subsets, not all characteristics. The subgroups' size can be selected. To select which class a new dataset belongs to, each decision tree assesses the data in its tree and classifies the data according to its predictions.

#### 2.2.5. Support Vector Machine (SVM)

This method classifies hyperplanes. SVM can perform regression and classification. This method's ideal plane separates the dataset into classes. Often, classifications are not as simple as a two-class situation. Classification often requires more complicated planes. The classifying plane of a two-class nonlinear issue is now a curve. In three dimensions, it is a curved plane. SVM is a good classification algorithm. SVM contains kernel function and margin ideas (range). Margin is the distance between nearest data support vectors and separation boundary. The SVM seeks to maximize this distance to solve a linearly separable problem. When data are not linearly separable, a kernel function is employed to project them onto a broader space.

#### 2.2.6. Boosting Methods and Gradient Boosting Machine Algorithm

Boosting a weak learning algorithm by majority [13] creates a strong algorithm from a linear combination of weak algorithms. The fact that these weak algorithms outperform random algorithms is enough to use them. The model created by applying algorithms to new data considers the linear combination of methods.

#### 2.2.7. Adaboost (Adaptive Boosting) Algorithm

The study used Adaboost [15]. Each stage creates a new estimated probability distribution on the learning data based on the preceding algorithm's results. The weights of the misclassified data are increased at each level. Thus, difficult-to-classify data can be focused on. We start with the most likely one of our learning algorithms. This algorithm teaches all data groupings a rule. Some actions are performed on the misclassified data to increase their weights, and the final state is used to classify the following algorithm. The weights of difficult-to-classify data increase towards the end of learning. Algorithms that classify accurately have their coefficients enhanced. So, their effects are amplified in the outcome hypothesis.

#### 2.2.8. Artificial Neural Networks

This program seeks to process information like the human brain. A brain's intricate network of linked neurons processes information. Diverse brain areas have different tasks for neurons. The network carries electrical signals between billions of neurons. Each neuron gets information through its “dentrid” region, alters it in its nucleus, and transfers it to the next neuron via its “axon” region. Synapses are the points where an axon meets a dendrite. Artificial neural networks also use connections between neurons. Neurons send signals to each other. It sends a signal to the next neuron by summing the signals.

### 2.3. Deep Learning

Deep learning, or deep artificial neural networks, is a subset of ANN. While there is a relationship between the input and output layers, the design is multilayered. The input data are calculated at each layer to produce an output. The layers of this structure are also neural networks. Each layer gets the previous layer's output as input and transfers the data to the next layer. The network structure has various factors that can generate different networks. These factors include the number of hidden layers, networks within each hidden layer, and neurons within each network. No one architecture solves all problems [17]. The hidden layers are those between the input and output layers. A learning system must be established to employ these numerous hidden levels effectively. Various approaches have been devised to utilize many layers effectively. One of these is the backpropagation algorithm. This study uses “multilayer perceptrons” for deep learning.

#### 2.3.1. Multilayer Perceptron (MLP) Neural Network

MLP, a feedforward neural network, is used in deep learning. The input layer does not take any action. In the middle layers, the results of the operations are transferred to the next layer. Intermediate layers are called hidden layers because their results cannot be observed directly.

### 2.4. Performance Evaluation Criteria

Accurate classification is important in performance appraisal, but it is not sufficient on its own. For example, we also look at which examples we misclassified, which ones we included in which class, and which we misclassified. Let us define these criteria and define the complexity matrix.

#### 2.4.1. Confusion Matrix

The complexity matrix [16, 17] contains the information between the prediction made by the algorithm and the actual situation as a result of the classification made by the applied algorithm. The values in this matrix are taken into account when evaluating the performance. One of the columns and rows of this matrix represents the actual situation, and the other is the prediction result. Following is the complexity matrix resulting from the classification for a two-class problem.

We explain the complexity matrix through the patient or healthy example as follows:

- True positive (TP): those who are truly unwell and have been labeled as such by the algorithm
- False positive (FP): the number of people who are not genuinely unwell but deemed so by the algorithm
- False negative (FN): the algorithm's percentage of genuinely ill people yet is deemed healthy
- True negative (TN): people who are not unwell but are still labeled as such by the algorithm

Equation (2) is the most important value used to measure the accuracy of measure and classification.

(2) $$\begin{array}{c} \text{Accuracy}=\frac{\text{TP}+\text{TN}}{\text{TP}+\text{TN}+\text{FP}+\text{FN}}. \end{array}$$

### 2.5. Feature Selection

The feature selection aims to find the subset containing the features most related to the problem among all features. This process is vital in areas with many features, like DNA fragments, where it is difficult to distinguish the important ones from the rest. Feature selection methods remove unnecessary features or noise. Very necessary (for solving the problem) and less necessary (for understanding some examples) attributes remain. Their study was the first to use gene expression correlation as a screening method for feature selection [18, 19]. Feature selection is an important data preprocessing technique. Here is a list of reasons for choosing an attribute. Savings: using a subattribute set with fewer variables saves resources. Increasing classification accuracy: removing unnecessary features improves classification accuracy. This also helps to understand the problem. Making the model simpler: a model with few features is easier to analyze. For example, many decision tree features lead to a complex model, whereas a small number of features prevent this. Fewer features mean faster learning. This reduces the learning time. When deciding which features to remove, consider the problem at hand and the desired outcome. Many of the attributes likely share similar information. In such cases, the attributes are redundant. Necessary or appropriate attributes are those that contain the most classification information. We cannot say which attribute is more important in machine learning because the requirements vary by subject. Conversely, we can discuss an attribute's direct or indirect necessity on a subject. Directly necessary attributes are those that have a direct effect on the outcome. Some attributes are not effective on their own, but they are effective on the result when combined. The selection process involves some strategies. These usually involve finding the smallest subset that outperforms the classification result before selecting the features. In the case of thousands of features such as a microarray, methods that perform both are used. For *n* attributes, there is a probability of 2^*n*^ − 1 subsets. This may be impossible in a multifeature set. For this reason, this process has been simplified by using some methods.

#### 2.5.1. Forward Selection

Starting from the empty set, the attribute that gives the best result is added first and then the attribute that gives the best result when added to the existing set is selected. If there is a threshold value, it can be stopped when it is reached, or there is no improvement in the classification result. Backward selection: it works in the opposite logic of forwarding selection. The least useful of all attributes are eliminated and stopped when a threshold value is reached. Bidirectional selection: it is a method based on both addition and subtraction.

The elimination steps in Figure 1 and the two feature elimination method in this work are based on the back-selection method. In both methods, the stopping criterion was taken as finding the best 50 criteria and the calculations are continued accordingly.

#### 2.5.2. Recursive Feature Elimination

It gradually eliminates some of the attributes, i.e., back-selection is applied. This elimination is decided as follows: attributes that do not distinguish between different classes should be eliminated. Here, to measure the adequacy of contribution, the currently available features must be weighted using a classification method. The cross-validation method is applied in the feature elimination process to increase the accuracy in selecting the best features. The elimination steps are repeated until the highest distinctive features remain. Classification accuracy or feature count limitation can be used to stop this method.

#### 2.5.3. Randomized Logistic Regression

This method works by subsampling the features and fitting an L1-penalty logistic regression. This method reduces attributes by disabling (punishing) unnecessary attributes. The random subsample selection process is repeated many times, and the features selected many times are selected as good features.

#### 2.5.4. *K*-Fold Cross-Validation (K-FCV)

For the classification result to be correct, the data used in learning should not be used for testing. To achieve this, cross-validation methods are applied. In the *k*-fold crossover method, the initial data are divided into *k* clusters. Each time, one of these clusters is reserved for testing and *k* − 1 for training. In this way, the study first determined [20, 21] that a realistic result would be reached by dividing the dataset into many parts. In this study, we split the data into five parts and then used a 5-fold crossover process, one piece at a time as testing and other pieces as training sets.

In the crossover method in Figure 2, the dataset is divided into ten parts. 9 of them are used to train the machine, and the rest are used for testing. Then, the same process was performed ten times, with all the pieces being the test set, respectively. In this work, a 5-fold crossover is used.

### 2.6. Backpropagation Algorithm

This algorithm first propagates data from the input to the output layer to obtain all outputs. Then, the hidden layers are returned to reduce the amount of error found. Each cycle reduces error by applying a process like a gradient reduction. The algorithm is stopped here by several iterations or an error rate. To optimize the differentiable and continuous function and to find the line on which it will make a little progress, this method first takes the partial derivative of the objective function according to the gradient calculation at a point. If the location is not optimal, it goes one step further using the same method. The algorithm stops once it finds it. The partial derivative of the objective function concerning the variables is all it takes to find the optimum quickly. Optimization is used in many areas. It is the process of selecting the best solution from a set of alternatives. It is still extensively researched and used. It is used in economics, modeling, error tracking, and data analysis. Other than optimization, many solutions can be proposed to these problems, but these solutions can only be applied under certain conditions. Many of these issues require extensive research to solve, which may not be feasible in a reasonable time frame. Data science processing and analysis of multidimensional data is an example. Too many variables are there in microarray datasets.

## 3. Results and Discussion

Seven classical machine learning methods were applied to the first breast cancer data with 133 samples with 1919 features and the second breast cancer data with 97 samples with 24481 features using Python language. While doing this, tests were performed without using any feature elimination method. According to this, logistic regression with 99.23% in the first data and the random forest method with 67.42% in the second data found the best results. Results found by other methods are also shown in the graphs on the following pages. The same dataset was then scaled down by applying the LTE method to keep the best 50 features. As a result, the SVM method in the first data with 99.23% found the best classification result with 88.82% in the second data. The results of other methods are also shown in the graph. Again, by applying the RLR feature selection method to the same dataset, size reduction was made to leave the best 50 features. As a result, the SVM method was the method with the highest accuracy with 99.23% in the first data and 87.87% in the second data.

### 3.1. Results Found in the First Data

First, no feature elimination method was applied to the data. The results in the first case are shown in Figure 3. First, seven machine learning methods were compared to 1919 attribute data with 133 samples, our first dataset, without applying any feature elimination method.

In Figure 3, it is seen that the logistic regression method has the highest results and the decision tree method has the lowest results; it is seen that the logistic regression method after RLR has a lower rate than the first case, the K-FCV algorithm has not changed, and the other five algorithms give better results and we can also see that the logistic regression algorithm gives lower results than the first case, the K-FCV is the same, and the other five methods give better results. According to all the results in Figure 4, the highest SVM with 98.98% and the lowest decision tree with 90.28% were classified. This time, SVM, one of the deep learning methods, was applied to the same dataset by using different numbers of hidden layers and different neurons in each layer.

The number of hidden layers used and the number of neurons in each layer is shown under each column in Figure 5.

In Figure 5, in cases where 15 or 30 neurons are used in one hidden layer and 15-15 neurons are used in two hidden layers, only three pieces of data were misclassified with 97.69% and the highest accuracy rate was achieved. The results of other cases are shown in the graph. In the data we used, it was seen that increasing the number of layers in deep learning did not increase the accuracy. For example, when arranging according to the number of 3-layered 15-10-5 neurons, the accuracy rate has been determined to be lower than the 2-layered 15-15, 15-30, and 30-60 cases or single-layered 30.15 cases. It was observed that the classification accuracy decreased again when the LTE method, which is one of the feature methods, was applied. In the case of 15-15 line-ups, the accuracy rate before elimination was 97.69%, but after this method was applied, the result decreased to 94.62%. Since there were 133 samples in the first dataset we used, deep learning results were not higher than classical machine methods.

### 3.2. Results Found in the Second Data

Our second dataset has 24481 attributes with 97 samples. In this dataset, again, without applying any feature elimination method in the first case, it was applied later, and the results were compared.

In Figure 6, all seven machine learning methods can be seen to classify this data with low accuracy before any feature elimination method. Accuracy rates of all algorithms have increased significantly compared to before feature elimination. SVM gave the best result with 87.87%, and it is seen that the accuracy rates of all algorithms have increased significantly compared to the first case. It is seen that the SVM method again classifies at the best rate.

On average, the highest SVM accuracy with 78.81% and the lowest decision tree accuracy with 63.39% were classified.

It is seen in Figure 8 that MLP did not achieve high results. When 30 neurons are used in a single hidden layer, we see that the best result is achieved with 68.72% and the worst result is achieved when 60 neurons are used. It is seen that using 15-15 or 15-30 neurons in two hidden layers gives better results than using 30-60 neurons. It is seen that the use of 3 hidden layers, 15-10-5, gives the 2^nd^ best result. Using the same number of hidden layers, it can be said that increasing the number of neurons decreases the result. On average, we can say that machine learning methods perform better on this small number of samples.

## 4. Conclusion

In our study, we focused on the analysis of gene expression data. Microarray technology has brought a new perspective to the field of cancer studies and diagnosis of diseases in general, but working with this type of data can be evaluated under large-scale optimization processes because gene expression data contain so much data that it can be expressed in the tens of thousands. Therefore, various methods have been developed and are being developed to analyze data in this dimension. Applications were made with supervised machine learning and deep learning techniques. These applications are the first data on breast cancer diagnosis and the second data on whether it will recur. The first of these data was used only in one study, and the other was used in many studies. Using these data was first used to perform machine learning. After processing the data first and applying the size reduction process, the prediction accuracy was compared with many methods. In the dimension reduction process, feature elimination was performed so that 50 best features remained. Algorithms were compared on both datasets before and after performing this operation. Higher results were achieved on the initial data. After the feature methods, the SVM method is classified with the highest accuracy and the decision trees with the lowest accuracy in both datasets. In addition, the same feature methods used in both datasets, LTE and RLR, gave close results in all algorithms. MLP gave close results in the first data with machine learning methods. The second data, on average, gave significantly lower results. It can be said that the small number of examples is effective in this result because a large number of examples is required for effective learning of MLP. In our data, the data numbers are 133 and 97. Since the first data are easy to classify, all methods have classified over 90% before and after feature elimination. The 2^nd^ data are difficult to classify, and the results before feature elimination are low. After the feature elimination methods, the classification rate increased significantly in all methods, mostly in SVM. Here, the importance of feature elimination methods is understood.

## Figures and Tables

**Figure 1:** Attribute elimination stages.

**Figure 2:** *K*-fold cross-validation method.

**Figure 3:** Results before feature selection, after the RLR feature selection method, and after the LTE feature elimination method.

**Figure 4:** All results before and after feature elimination.

**Figure 5:** Results of deep learning by different layers.

**Figure 6:** Results before feature elimination in the 2^nd^ data, by applying RLR to 2^nd^ data, and by HT application to 2^nd^ data.

**Figure 7:** All results before and after feature elimination in the 2^nd^ data.

**Figure 8:** Results of deep learning in 2nd data by different layers.

## Data Availability

The data used to support the findings of this study are included within the article.
